# The Effect of Oxytocin plus Carboprost Methylate in Preventing Postpartum Hemorrhage in High-Risk Pregnancy and Its Effect on Blood Pressure

**DOI:** 10.1155/2022/9878482

**Published:** 2022-05-30

**Authors:** Lin Wei, Haiping Yang, Xiaoli Sun

**Affiliations:** Department of Obstetrics, Anhui Lujiang County People's Hospital, Lujiang County, Lucheng, Anhui Province, China

## Abstract

*Objective*. This study aimed to explore and analyze the effectiveness of oxytocin plus carboprost methylate in preventing postpartum hemorrhage in high-risk pregnancies and its effect on blood pressure. A total of 60 women with high-risk pregnancies who gave birth in our hospital from January 2020 to May 2021 were recruited and assigned via random number table method (1 : 1) to receive either oxytocin (control group) or oxytocin plus carboprost methylate (observation group). Outcome measures included hemorrhage and blood pressure. The bleeding volume of the women in the observation group (210.55 ± 45.98, 45.21 ± 9.27, and 73.74 ± 12.18) was significantly less than that in the control group during delivery and 2h and 24h after the delivery (276.91 ± 49.21, 72.98 ± 19.68, and 92.61 ± 15.67) (all *P* < 0.05). The observation group showed a significantly lower bleeding rate (6.67%) than the control group (16.67%) (*P* < 0.05). The two groups showed similar diastolic and systolic blood pressures (*P* > 0.05). Oxytocin plus carboprost methylate suppository effectively prevents postpartum hemorrhage in high-risk pregnancies, significantly reduces the amount of postpartum hemorrhage in high-risk pregnancies, and has little effect on the blood pressure of patients. Given its favorable treatment efficiency and high safety profile, this treatment protocol shows great potential for clinical application.

## 1. Introduction

High-risk pregnancies refer to pregnancies that involve increased health risks for the mother, the fetus, or both, with a significantly higher maternal and neonatal morbidity and mortality versus normal pregnancies [1]. Women with high-risk pregnancies are vulnerable to pregnancy complications such as high blood pressure, gestational diabetes, and preterm labor, which necessitate intensive care to enhance the health of the mother and the fetus [2]. Postpartum hemorrhage [3] is heavy vaginal bleeding (500 ml or more) within 24 hours after delivery. It is a serious complication during delivery and accounts for 25% of maternal deaths in China [4, 5]. The main causes of postpartum hemorrhage include uterine atony, detrimental placental profiles, perineal laceration, and coagulation dysfunction [6]. Studies have found that high-risk pregnancies are associated with a significantly higher postpartum hemorrhage rate compared with normal pregnancies, and postpartum hemorrhage may result in hemorrhagic shock, disseminated intravascular coagulation, and even maternal death [7, 8]. Oxytocin [9] is a peptide hormone secreted by the posterior pituitary and synthesized by the paraventricular and supraoptic nuclei of the hypothalamus [10]. It stimulates lactation, promotes the contraction of uterine smooth muscle during delivery, and lowers stress hormone levels such as adrenaline, thereby lowering blood pressure [11, 12]. Carboprost methylate [13] is a derivative of natural prostaglandin F2*α* and is widely present in various tissues and body fluids. It increases the frequency and amplitude of uterine contractions and enhances the contractility of uterine muscle, thereby promoting uterine contractions. At present, research has reported that carboprost methylate suppository avoided laborious treatment procedures and effectively reduced the amount of postpartum hemorrhage with manageable safety [14]. Therefore, by comparing the effectiveness of oxytocin mono-therapy versus combined therapy of oxytocin plus carboprost methylate, this study was to explore and analyze the effect of oxytocin combined with carboprost methylate in preventing postpartum hemorrhage in high-risk pregnancies and its effect on blood pressure, so as to provide a basis for clinical treatment. The research results are as follows.

## 2. Materials and Methods

### 2.1. Study Design and Participants

In this prospective, randomized, controlled study, 60 women with high-risk pregnancies who gave birth in our hospital from January 2020 to May 2021 were selected and assigned via random number table method to an observation group (*n* = 30). This project was reviewed and approved by the Research Ethics Committees of Anhui Lujiang County People's Hospital, No. AH9647.

### 2.2. Inclusion and Exclusion Criteria

#### 2.2.1. Inclusion Criteria

Patients who met the diagnostic criteria for high-risk pregnancy in Obstetrics and Gynecology, with one or more high-risk factors for postpartum hemorrhage [15], and who provided written informed consent were included.

#### 2.2.2. Exclusion Criteria

Patients with allergies to the drugs used in this study with psychiatric diseases, with relevant contraindications, and with hospital referral or withdrawal of consent were excluded.

### 2.3. Methods

Both groups were admitted to our hospital before delivery. The women in the control group received 20 U of oxytocin (Beijing Saisheng Pharmaceutical Co., Ltd., National Pharmacopoeia H11020363) through intramuscular injection immediately after delivery. A similar administration regimen of oxytocin was introduced to those in the observation group.

Except for oxytocin administration, the women in the observation group one also received carboprost methylate suppository (Northeast Pharmaceutical Group Shenyang No.1 Pharmaceutical Co., Ltd. State Drug Quantiėer H10800006). The midwife placed the carboprost methylate suppository in 1/3 part of the anterior vaginal wall and kept it there for 2 min until the suppository dissolved to avoid a decrease in the efficacy of the suppository as it might be displaced by the blood flow. If bleeding persisted, the drug was administered through the anus.

### 2.4. Evaluation Criteria

1. The blood loss in the two groups of patients during delivery, 2 hours after the delivery, and 24 hours after the delivery was recorded. The volume of blood in the blood collector and in the gauze after delivery was recorded separately using a combination of the volumetric method and area method. The volume of gauze blood was estimated according to the wet area of gauze blood, and the actual amount of bleeding at delivery was calculated as the sum of the two. The postpartum bleeding volume at 2 h and 24 h was recorded by weighing the weight of the mattress, and the actual bleeding volume was accurately calculated and compared between groups.
2. The number of bleeding cases within 2 hours and 24 hours after the delivery was recorded, and the bleeding rates were calculated for comparison.
3. The blood pressure of the two groups of women before and after treatment was recorded, and the systolic blood pressure and diastolic blood pressure of the two groups of women before and after the treatment were continuously monitored and compared.

### 2.5. Statistical Analysis

All data analyses were performed with SPSS22.0 software. Enumeration data are expressed as [n (%)] and analyzed using the chi-square test, and measurement data are expressed as (mean ± SD) and analyzed using the t-test. Differences were considered statistically significant at *P* < 0.05.

## 3. Results

### 3.1. General Data

The women in the observation group were aged 21–42 years, with a mean age of 28.53 ± 5.32 years, and the gestational week was 34-42 weeks, with a mean of 39.08 ± 2.18 weeks. The women in the control group were aged 19–37 years, with a mean age of 28.64 ± 4.54 years, and the gestational week was 34–42 weeks, with a mean of 39.23 ± 1.99 weeks. There were no significant differences in general data between the two groups (Table 1).

### 3.2. Bleeding

#### 3.2.1. Bleeding Volume

The bleeding volume of the women in the observation group (210.55 ± 45.98, 45.21 ± 9.27, and 73.74 ± 12.18) was significantly less than that in the control group during delivery and 2 h and 24 h after the delivery (276.91 ± 49.21, 72.98 ± 19.68, and 92.61 ± 15.67) (all *P* < 0.05) (Table 2).

#### 3.2.2. Number of Bleeding Cases

The bleeding rate of the observation group (6.67%) was significantly lower than that of the control group (16.67%) (*P* < 0.05) (Table 3).

### 3.3. Blood Pressure

The differences in diastolic and systolic blood pressure in the observation group (85.87 ± 8.01, 122.12 ± 10.65/89.17 ± 6.12, 127.62 ± 11.28) and the control group (85.02 ± 7.98, 123.61 ± 10.17/89.68 ± 6.58, 126.88 ± 11.61) before and after treatment were not statistically significant (*P* > 0.05) (Table 4).

## 4. Discussion

The morbidity and mortality of pregnant women and newborns in high-risk pregnancies are significantly higher than those in normal pregnancies. Therefore, pregnancy tests are of great significance to achieve early prevention of high-risk pregnancies. Postpartum hemorrhage is a common obstetric complication and one of the main causes of maternal death. Previous literature results show that postpartum hemorrhage is predominantly attributed to complications elicited by high-risk pregnancies [16]. In addition, a cesarean section may result in more severe postpartum hemorrhage than natural childbirth [17]. Oxytocin promotes the contraction of the uterus, and estrogen can increase the sensitivity of the uterus to oxytocin, while progesterone is the opposite [18]. Carboprost methylate suppository is a prostaglandin uterine stimulant and is mainly used to prevent and treat postpartum hemorrhage caused by uterine atony [19], with a longer half-life of 30 min versus that of 3-4 min of oxytocin. It is metabolized and excreted in urine 6–9 h after administration, and the synergistic effect of carboprost methylate with oxytocin can effectively achieve postpartum hemorrhage control [20].

The results of the present study showed that the bleeding volume of the patients in the observation group was significantly less than that of the patients in the control group, and the bleeding rate of the observation group was significantly lower than that of the control group, suggesting that oxytocin plus carboprost methylate suppository effectively prevented or mitigated postpartum hemorrhage in patients. The reason may be that oxytocin promotes the contraction of uterine smooth muscle during childbirth. The sensitivity of the uterine to oxytocin is closely related to the levels of estrogen and progesterone in the body, and the effect of uterine contractions enhancement is less obvious with a dose of more than 40 U. Carboprost methylate enhances the frequency and amplitude of uterine contractions and is in use with oxytocin; however, the duration of efficacy is short, which requires cautious use. Research has shown that improper use of carboprost methylate is associated with prolonged incision and amniotic fluid embolism, causing reflex contractions of the uterus and increased bleeding. Therefore, the use of oxytocin in combination with carboprost methylate suppositories at different timings can compensate for the deficiencies in the onset of action and half-life. The combined use of the two better exerts the drug effect and effectively prevents cesarean section and postoperative bleeding. The results of the present study also showed that the diastolic blood pressure of the observation group and the control group before and after treatment showed no significant differences, suggesting that the two methods had little effect on the blood pressure of patients, because oxytocin reduces the levels of stress hormones such as adrenal ketone in the human body, while carbamide had no effect on the blood pressure, pulse, and oxygen saturation. However, due to the limited sample size of this study, follow-up studies are still needed.

## 5. Conclusion

Oxytocin combined with carboprost methylate suppository effectively prevents postpartum hemorrhage in high-risk pregnancy, significantly reduces the amount of postpartum hemorrhage in high-risk pregnancy, and has little effect on the blood pressure of parturient women.

## Figures and Tables

**Table 1:** Comparison of general data of the two groups of patients ($\bar{x}\pm s$).

Groups	*n*	Age	Gestational age
Observation group	30	28.53 ± 5.32	39.08 ± 2.18
Control group	30	28.64 ± 4.54	39.23 ± 1.99
*t*		0.086	0.278
*P*		0.932	0.782

**Table 2:** Comparison of bleeding volume between two groups of patients ($\bar{x}\pm s$).

Groups	*n*	Intraoperative blood loss	2 h postoperative bleeding	24 h postoperative bleeding
Observation group	30	210.55 ± 45.98	231.21 ± 25.27	259.74 ± 32.18
Control group	30	303.91 ± 49.21	372.98 ± 39.68	392.61 ± 35.67
*t*	—	7.593	15.506	15.149
*P*	—	<0.001	<0.001	<0.001

**Table 3:** Comparison of bleeding rates between the two groups of patients (%).

Groups	n	No bleeding	Bleeding	Bleeding rate
Observation group	30	28	2	6.67
Control group	30	25	5	16.67
*x* ^2^	—			1.456
*P*	—			0.022

**Table 4:** Comparison of blood pressure levels in the two groups before and after treatment ($\bar{\text{x}}$ ±s).

Groups	*n*	Before treatment		After treatment	
		DBP	SBP	DBP	SBP
Observation group	30	85.87 ± 8.01	122.12 ± 10.65	89.17 ± 6.12	127.62 ± 11.28
Control group	30	85.02 ± 7.98	123.61 ± 10.17	89.68 ± 6.58	126.88 ± 11.61
*t*	—	0.412	0.554	0.311	0.250
*P*	—	0.682	0.582	0.757	0.803

DBP, Diastolic Blood Pressure; SBP, Systolic Blood Pressure.

## Data Availability

The data generated or analyzed during this study are included within the article.
